The article "Jacarelhyperol A induced apoptosis in leukaemia cancer cell through inhibition the activity of Bcl-2 proteins" was retracted in 2022. Reasons: duplicated images; original data or images not available; unreliable results or conclusions.

# Jacarelhyperol A induced apoptosis in leukaemia cancer cell through inhibition the activity of Bcl-2 proteins

**DOI:** 10.1186/1471-2407-14-689

**Published:** 2014-09-22

**Authors:** Shoude Zhang, Jun Yin, Xia Li, Jigang Zhang, Rongcai Yue, Yanyan Diao, Honglin Li, Hui Wang, Lei Shan, Weidong Zhang

**Affiliations:** School of Pharmacy, Second Military Medical University, 325# Guohe Road, Shanghai, 200433 China; Shanghai Key Laboratory of New Drug Design, State Key Laboratory of Bioreactor Engineering, School of Pharmacy, East China University of Science and Technology, 130# Meilong Road, Shanghai, 200237 China; Key Laboratory of Nutrition and Metabolism, Institute for Nutritional Sciences, Shanghai Institutes for Biological Sciences, Chinese Academy of Sciences, Graduate School of the Chinese Academy of Sciences, 320# YueYang Road, Shanghai, 201203 China

**Keywords:** Bcl-2, Jacarelhyperol A, Apoptosis, *Hypericum japonicum* Thunb.ex Murray, Leukemia

## Abstract

**Background:**

*Hypericum japonicum* Thunb. ex Murray is widely used as an herbal medicine for the treatment of hepatitis and tumours in China. However, the molecular mechanisms of its effects are unclear. Our previous research showed that extracts of *H. japonicum* can induce apoptosis in leukaemia cells. We also previously systematically analysed and isolated the chemical composition of *H. japonicum*.

**Methods:**

The fluorescence polarisation experiment was used to screen for inhibitors of Bcl-2 proteins which are proved as key proteins in apoptosis. The binding mode was modelled by molecular docking. We investigated the proliferation attenuating and apoptosis inducing effects of active compound on cancer cells by MTT assay and flow cytometry analysis. Activation of caspases were tested by Western blot. A broad-spectrum caspase inhibitor Z-VAD-FMK was used to investigate the caspases-dependence. In addition, co-immunoprecipitation was performed to analyse the inhibition of heterodimerization between anti-apoptotic Bcl-2 proteins with pro-apoptotic proteins. Moreover, in vivo activity was tested in a mouse xenograph tumour model.

**Result:**

Jacarelhyperol A (Jac-A), a characteristic constituent of *H. japonicum*, was identified as a potential Bcl-2 inhibitor. Jac-A showed binding affinities to Bcl-x_L_, Bcl-2, and Mcl-1 with K_i_ values of 0.46 μM, 0.43 μM, and 1.69 μM, respectively. This is consistent with computational modelling results, which show that Jac-A presents a favorable binding mode with Bcl-x_L_ in the BH3-binding pocket. In addition, Jac-A showed potential growth inhibitory activity in leukaemia cells with IC_50_ values from 1.52 to 6.92 μM and significantly induced apoptosis of K562 cells by promoting release of cytochrome c and activating the caspases. Jac-A also been proved that its effect is partly caspases-dependent and can disrupt the heterodimerization between anti-apoptotic Bcl-2 proteins with pro-apoptotic proteins. Moreover, Jac-A dose-dependently inhibited human K562 cell growth in a mouse xenograph tumour model with low toxicity.

The article "Jacarelhyperol A induced apoptosis in leukaemia cancer cell through inhibition the activity of Bcl-2 proteins" was retracted in 2022. Reasons: duplicated images; original data or images not available; unreliable results or conclusions.

**Conclusion:**

In this study, a characteristic constituent of *H. japonicum*, Jac-A, was shown to induce apoptosis in leukaemia cells by mediating the Bcl-2 proteins. Therefore, we propose a new lead compound for cancer therapy with a low toxicity, and have provided evidence for using *H. japonicum* as an anti-cancer herb.

**Electronic supplementary material:**

The online version of this article (doi:10.1186/1471-2407-14-689) contains supplementary material, which is available to authorized users.

## Background

The entire *Hypericum japonicum* herb, named “Tianjihuang,” is widely used for the treatment of infectious hepatitis, acute and chronic hepatitis, and tumour in China [1]. An 85% ethanol-treated water extract is documented in the Chinese Pharmacopoeia as an injection for the treatment of viral hepatitis [2, 3]. Moreover, *H. japonicum* is used as an animal feed in China because of its widespread growth. These records demonstrate the clinical safety of *H. japonicum*. However, the molecular mechanisms of its effects are unclear. To better understand the mechanisms of *H. japonicum*, its chemical composition was systematically isolated and analysed in our previous study. In this study, we identified jacarelhyperol A (Jac-A), a characteristic constituent of *H. japonicum*, as a potent inhibitor of Bcl-2 proteins *via* high throughput screening of an in-house natural product library (NPL).

The Bcl-2 family of proteins play an important role in apoptosis through the balance of antiapoptotic proteins (e.g., Bcl-2, Bcl-x_L_, Mcl-1) and proapoptotic proteins (e.g., Bak, Bax, Bad, Bid) [4]. The ability of antiapoptotic proteins to form heterodimers with a number of proapoptotic proteins is believed to play a crucial role in their antiapoptotic function [5]. Antiapoptotic Bcl-2 proteins are overexpressed in a variety of tumours, which can protect cancer cells from apoptosis [6, 7]. Owing to their important functions in regulating cell death, the pharmacological inhibition of Bcl-2 proteins is a promising strategy for apoptosis induction or sensitisation to chemotherapy [8]. Protein sequence analysis and structure-function studies revealed that the BH3 domain of proapoptotic proteins is the fundamental motif for the dimerisation with antiapoptotic proteins [9]. The three-dimensional structure of a complex of Bcl-x_L_ and the Bak BH3 domain peptide showed that the Bak peptide is an amphipathic α-helix that binds to a hydrophobic groove on the surface of Bcl-x_L_ [10]. Based on these studies, screening new ligands that bind to the same pocket became an anti-cancer drug discovery strategy to search for antiapoptotic protein inhibitors [11]. To screen for Bcl-2 protein inhibitors, we used fluorescence polarisation (FP), whose basic principle is that a fluorescent peptide tracer (Flu-Bid-BH3) and a nonfluorescent small molecule inhibitor compete for binding to the Bid BH3 domain of Bcl-2 proteins. Jac-A was chosen as the candidate compound for further research because of its high affinity with Bcl-2 proteins and favorable binding mode with Bcl-x_L_. Then, we tested its anti-cancer activity *in vitro* and *in vivo*. Jac-A possesses a broad antitumour effect for all tested cancer cells and remarkably inhibited the proliferation of leukaemia cells. Moreover, Jac-A not only induced K562 cell apoptosis *in vitro*, but also inhibited human K562 cell growth in a mouse xenograph tumour model, which provided evidence for using *H. japonicum* as an anti-cancer herbal medicine. We also proved that Jac-A’s effect is partly caspase-dependent and it can disrupt the heterodimerization between anti-apoptotic Bcl-2 family members with pro-apoptotic Bcl-2 family members.

The article "Jacarelhyperol A induced apoptosis in leukaemia cancer cell through inhibition the activity of Bcl-2 proteins" was retracted in 2022. Reasons: duplicated images; original data or images not available; unreliable results or conclusions.

## Methods

### Fluorescence polarisation assay

The Bid BH3 domain peptide (sequence: EDIIRNIARHLAQVGDSMDR) was synthesised and labelled with 5-Carboxyfluorescein (5-FAM) at the N-terminus. For the competitive binding assay, 200 nM Bcl-x_L_, Bcl-2, or Mcl-1 was mixed with various concentrations of compounds in PBS (4.3 mM Na_2_HPO_4_, 1.4 mM KH_2_PO_4_, 137 mM NaCl, 2.7 mM KCl, pH 7.4). After incubation for 1 h at 37°C, an equal volume of 200 nM 5-FAM-labelled BH3 peptide was added to the solution. After incubation for 10 min at 37°C, the fluorescence polarisation was measured on a TECAN Genios Pro microplate reader. The excitation wavelength and emission wavelength were set to 485 nm and 535 nm, respectively. The 50% inhibiting concentration (IC_50_) value was analysed by the GraphPad Prism program. The Ki was calculated by a web-based tool [12].

### Molecular modelling

The refined structure of Bcl-x_L_ (PDB: 2YXJ) was used for prediction binding mode between Jac-A with Bcl-x_L_. The program Maestro 9.0 was used for this assessment. All water molecules were removed from the structure of the complex. Hydrogen atoms and charges were added during a brief relaxation that was performed using the “Protein Preparation Wizard” workflow in Maestro 9.0. After optimising the hydrogen bond network, the crystal structure was minimised using the OPLS 2005 force field with the maximum root mean square deviation (RMSD) value of 0.3 Å. The grid-enclosing box was centred on the ligand ABT-737 in the refined crystal structure as described above, and defined so as to enclose the residues located within 14 Å from the ligand. This domain has been identified as the BH3 domain, which is the fundamental motif for dimerization with the BH3 peptide. The three-dimensional structure of Jac-A was generated with the Ligprep module. Docking process was performed using GLIDE with default docking parameter setting with extra precision (XP) approach.

The article "Jacarelhyperol A induced apoptosis in leukaemia cancer cell through inhibition the activity of Bcl-2 proteins" was retracted in 2022. Reasons: duplicated images; original data or images not available; unreliable results or conclusions.

### Cell culture

Cell lines MBA-MB-231, T47D, LOVO, A549, HepG2, K562, HL-60, and THP-1 cells were obtained from the American Type Culture Collection (Manassas, VA). All cell culture supplies were obtained from Invitrogen (Carlsbad, CA). Thiazolyl blue tetrazolium bromide (catalogue no. M5655) and dimethyl sulfoxide (catalogue no. D5879) were purchased from Sigma-Aldrich (St. Louis, MO). Cells were cultured in RPMI 1640 (A549, K562, THP-1), IMDM (HL-60), or DMEM (MBA-MB-231, LOVO, T47D, HepG2) and maintained in a Thermo incubator (Waltham, MA) with humidified air containing 5% CO_2_ at 37°C. All culture media contained 10% FBS and 1% penicillin-streptomycin.

### Cytotoxicity assay

The cytotoxic activitiy of Jac-A against human cancer cells was measured by the MTT colorimetric assay. Four thousand cells (per well) were seeded in 96-well plates and treated with the compounds for 48 h at serial concentrations. Then, 10 μL MTT solution (5 mg/mL in PBS) was added to each well, and the plates were incubated for an additional 2–4 h at 37°C. The supernatant was carefully removed, and 100 μL DMSO was added to dissolve the formazan crystals. The absorbance at 570 nm was recorded on a BioTek Synergy 2 plate reader (BioTek Instruments, Inc., Winooski, Vt, USA).

### Detection of apoptosis by flow cytometry using Annexin V-PI staining

After treated with 0 (control), 0.1, 1, 5, 10 μM/L Jac-A and 0.5% DMSO for 48 h, K562 cells from each group were collected and diluted to a concentration of 1.0 × 10^6^ per mL. The cells were washed with cold PBS twice and resuspended in 100 μL Annexin-V-FITC (Sigma) diluted 1:100 in binding buffer (10 mM Hepes 100 mM NaCl, 10 mM KCl, 1 mM MgCl_2_, 1.8 mM CaCl_2_) containing 10% propidium iodide (PI, Sigma) for 30 min at 4°C. The apoptosis were detected by Flow Cytometry (BD Biosciences).

### Cytochrome c release assay

The method of preparing mitochondria and cytosol was referenced to others [13–15]. Briefly, after treated with 0 (control), 3, 6, 12 μM/L Jac-A for 48 h, K562 cells (1 × 10^6^) were collected and washed once with ice-cold PBS and re-suspended in mitochondrial isolation buffer (250 mM sucrose, 20 mM HEPES, pH 7.4, 5 mM MgCl2 and 10 mM KCl ) containing 0.05% digitonin. Cells were left on ice for 10 min followed by centrifugation at 13000 r.p.m. for 3 min. The pellete was the mitochondrial membrane (heavy membrane proteins) portion. Soluble fraction proteins and an equivalent amount of heavy membrane proteins were subjected to SDS-PAGE and analysed by Western blot with antibodies against Cyt c (Abcam, CA).

The article "Jacarelhyperol A induced apoptosis in leukaemia cancer cell through inhibition the activity of Bcl-2 proteins" was retracted in 2022. Reasons: duplicated images; original data or images not available; unreliable results or conclusions.

### Caspase activation assay by western blotting

After treated with 0 (control), 3, 6, 12 μM/L Jac-A for 48 h, K562 cells (1 × 10^6^) were collected and suspended in lysis buffer containing 150 mM NaCl, 50 mM Tris (pH 8.0), 0.02% NaN_3_, 0.01% PMSF, 0.2% Aprotinin, and 1% TritonX-100 supplemented with protease inhibitor cocktail (Thermo Scientific). Fifty micrograms protein per lane was electrophoresed on 10% SDS polyacrylamide gels. Nonspecific reactivity was blocked by 5% non-fat milk prepared in TBST (10 mM Tris, 150 mM NaCl, 0.05% Tween-20, pH 7.5) at room temperature for 1 h. The membranes were incubated with antibodies diluted according to the manufacturers’ instructions. Images were captured by the Odyssey infrared imaging system (Li-Cor Bioscience, Lincoln, NE). Protein densitometry was performed with the Quantity One imaging software (Bio-Rad) and normalised against β-actin. Antibodies for cleaved PARP, PARP, cleaved caspase-9, caspase-9, cleaved caspase-3, caspase-3, and β-actin were obtained from Cell Signaling Technology (Beverly, MA).

### Co-immunoprecipitation

Immunoprecipitation was prepared as the method reported by others [14, 16]. After treated with 0 (control), 3, 6, 12 μM/L Jac-A for 48 h, K562 cells (1 × 10^6^) were collected and suspended in CHAPS (3-[(3-cholamidopropyl) dimethylammonio]- 1-propansulfonate) lysis buffer containing 150 mM NaCl, 10 mM HEPES [pH 7.4], 1% CHAPS, 1 mM PMSF, 5 μg/ml leupeptin, 5 μg/ml aprotin and 1 μg/ml pepstain A. 150 μg of K562 cell lysates in 500 μL of CHAPS lysis buffer were precleared for 60 min at 4°C with 20 μL of a 1:1 slurry of protein A/G Plus-Agarose (Santa Cruz Biotechnology, Cat.# sc 2003) and 1 μg of rabbit IgG. After a brief centrifugation (3000 × g for 5 min at 4°C) to remove precleared beads, 1 μg of rabbit anti-Bax or Bakpolyclonal antibody and 20 μL of Protein G Plus-Agarose were added to the lysate, followed by incubation at 4°C overnight on a rotating device, precipitates were washed four times with CHAPS buffer, resuspended in 30 μL 1× SDS electrophoresis sample buffer (50 mM Tris–HCl (pH 6.8), 100 mM dithiothreitol, 2% SDS, 0.1% bromophenol blue, and 10% glycerol), electrophoresed, and analysed by Western blotting with monoclonal antibodies against Bcl-x_L_, Bcl-2, Mcl-1, Bax, and Bak, respectively. All antibodies in this experiment were purchased from Abcam (Shanghai, CA)

The article "Jacarelhyperol A induced apoptosis in leukaemia cancer cell through inhibition the activity of Bcl-2 proteins" was retracted in 2022. Reasons: duplicated images; original data or images not available; unreliable results or conclusions.

### Xenograph tumor model in mice

Female Balb/c nude mice (5 weeks old) were purchased from Shanghai SLAC Laboratory Animal Co., LTD (Shanghai, China). 5 × 10^6^ K562 cells were subcutaneously injected in the right flank of mice. When the tumours reached approximately 200 mm^3^, the mice were randomly divided into four groups (n = 10 mice/each group) and treated with Jac-A at 2, 10, 50 mg/kg or vehicle by oral gavage. Tumour growth was monitored by measuring the tumour size twice a week for 3 weeks after treatment. A digital calliper was used to measure the tumour in two orthogonal dimensions. The volume was calculated with the formula (long dimension) × (short dimension)^2^/2. The body weight and survival of the nude mice were monitored throughout the experiments. All animal experiments were approved by the animal care committee of the Second Military Medical University in accordance with institutional and Chinese government guidelines for animal experiments.

### Statistical analysis

The data from the *in vitro* and *in vivo* experiments at different time points for the different treatment groups were analysed for statistical significance with the GraphPad Prism program (GraphPad, San Diego, CA). One-way ANOVA was used among groups, followed by the Mann–Whitney *U* test for post hoc comparisons to determine the *P* values. The statistical significance of differences in the survival of mice from the different groups was determined by the log-rank test using the same program.

### Chemistry

The purity of Jac-A was verified with NMR and HPLC, and the purity of Jac-A was 97%. *Jacarelhyperol A* [17], isolated from *Hypericum japonicum* Thunb.ex Murray; yellow powder; ^1^H-NMR (DMSO-*d*_*6*_, 500 MHz, *δ*_H_): 6.78 (1H, d, *J* = 10 Hz), 5.86 (1H, d, *J* = 10 Hz), 7.63 (1H, d, *J* = 8 Hz), 7.03 (1H, d, *J* = 8 Hz), 7.51 (1H, d, *J* = 8 Hz), 6.92 (1H, d, *J* = 8 Hz), 6.29 (1H, s); ^13^C-NMR (DMSO-*d*_*6*_, 125 MHz, *δ*_C_): 70.2, 71.0, 78.4 (×2), 79.2, 97.6, 98.6, 100.7 (×2), 101.4, 102.6, 102.9, 112.8, 113.0, 113.7 (×4), 115.7, 116.8, 128.2 (×2), 131.6, 132.7, 145.4, 145.9, 149.6, 151.0 (×2), 151.9, 159.8, 162.3, 162.8, 179.7 (×2), 179.9; ESIMS: *m/z* 667 [M - H]^-^; (-)-Gossypol (98% purity) was purchased from Sigma–Aldrich (Shanghai, CA)

## Results

### Screening active compounds

Fuoresence polarization was used to screen for Bcl-2 protein inhibitors. Jac-A was chosen as the candidate compound for further research because of its high affinity to Bcl-2 proteins. As shown in Figure 1 and Table 1, Jac-A can dose-dependently bind to Bcl-x_L_, Bcl-2, and Mcl-1 with a K_i_ value of 0.46 μM, 0.43 μM, and 1.69 μM, respectively, which near to the activity of positive control (-)-Gossypol, a known Bcl-2 protein inhibitor.

The article "Jacarelhyperol A induced apoptosis in leukaemia cancer cell through inhibition the activity of Bcl-2 proteins" was retracted in 2022. Reasons: duplicated images; original data or images not available; unreliable results or conclusions.

**Figure 1:** **The inhibitory activity of Jac A to Bcl-2 proteins. (A)** The structure of Jac A. **(B)** The inhibitory curves of Jac-A to Bcl-x_L_, Bcl-2, and Mcl-1 by fuoresence polarization. The substrate for the assay was a 5-FAM-labeled Bid BH3 domain peptide (amino sequence: EDIIRNIARHLAQVGDSMDR).

**Table 1:** **Binding affinity of Jac-A and (-)-gossypol with Bcl-x**_**L**_ **, Bcl-2 or Mcl-1 determined by a fluorescence polarisation assay (Ki, μM)**

Compound	Bcl-x _L_	Bcl-2	Mcl-1
**Jac-A**	0.46	0.43	1.69
**(-)-Gossypol**	1.01	0.95	0.86

### Predicting the binding modes of Jac-A with Bcl-x_L_

To map the binding site of Jac-A, we built complex structure of the compound with Bcl-x_L_ by docking (Figure 2). Jac-A contains two xanthones and can generates many conformations by rotating the C10 - O and O - C3″ bonds. The best binding model is shown in Figure 2A, in which the two xanthones of Jac-A exhibit two different orientations with a 90° dihedral angle and occupy three sub-pockets (P2, P4, and P5). The three sub-pockets play an important role in binding with pro-death BH3-only proteins and ligands. The P2 pocket, formed by residues Tyr-101, Ala-104, Leu-108, Val-126, Asn-135, Ala-142, and Ser-145, makes hydrophobic contacts with the aromatic H ring of Jac-A. In the P4 pocket, the aromatic B ring, double bond of the A ring, and the two methyl groups at C-3 make hydrophobic contacts with the hydrophobic pocket formed by residues Glu-96, Phe-97, Gly-138, and Tyr-195. Moreover, the hydrophobic group D ring and isopropyl at C-2″ of Jac-A can generate a hydrophobic interaction with the P5 pocket formed by residues Leu-130, Arg-132, and Arg-139. In addition, the three hydroxyl groups of Jac-A are predicted to form a hydrogen bond with the polar atoms of residues Gly-138, Tyr-101, and Glu-129 (Figure 2B).

**Figure 2:** **The predicted binding mode of Jac-A in the binding site of Bcl-x**_**L**_ **(PDB code 2YXJ). (A)** The binding site and orientation of Jac-A in the hydrophobic groove of Bcl-x_L_. Jac-A occupies three key sub-pockets (P2, P4, and P5) which play an important role in binding with pro-death BH3-only proteins and ligands. The protein is rendered in green, while the compound is rendered in purple. The P2, P4, and P5 binding pockets are labelled with dash circles. **(B)** The interaction model between Jac-A with Bcl-x_L_. Jac-A can form three hydrogen bonds with the polar atoms of residues Gly-138, Tyr-101, and Glu-129. Bcl-x_L_ is rendered as a cartoon, while the residues in contact with the ligand and compound are rendered as sticks. The residues are rendered in green, and the compound is coloured in purple. The hydrogen bonds are represented by dotted black lines.

The article "Jacarelhyperol A induced apoptosis in leukaemia cancer cell through inhibition the activity of Bcl-2 proteins" was retracted in 2022. Reasons: duplicated images; original data or images not available; unreliable results or conclusions.

### Anti-cancer activity of Jac-A

Bcl-x_L_, Bcl-2, and Mcl-1 are overexpressed in multiple cancer cells and contribute to tumour drug resistance [18]. Since Jac-A binds to Bcl-x_L_, Bcl-2, and Mcl-1 with high affinity and inhibits their interactions with the BH3 domain of proapoptotic proteins, we elected to study the effect of Jac-A on cancer cells. Using the MTT assay, we tested the cytotoxicity of Jac-A against various human cancer cell lines. Remarkably, Jac-A induced a dose-dependent reduction in cell viability compared to positive control doxorubicin (Table 2). Jac-A exhibited cytotoxic potency against breast cancer cells (MBA-MB-231, T47D), colon cancer cells (LOVO), lung cancer cells (A549), liver cancer cells (HepG2), and leukaemia cancer cells (K562, HL-60, THP-1). Jac-A showed strongest activity against leukaemia cells with IC_50_ values from 6.52 to 9.92 μM. Our results demonstrate that Jac-A possesses broad anti-cancer effects.

**Table 2:** **The inhibitory activity of Jac-A on tumour cells** ***via*** **MTT Assay (IC**_**50**_ **,** ***μ*** **M, n = 4, mean ± SD)**

Compound	Breast cancer		Colon cancer	Lung cancer	Liver cancer	Leukaemia		
	MBA-MB-231	T47D	LOVO	A549	HepG2	K562	HL-60	THP-1
Jac-A	**22.61 ± 1.2**	**12.53 ± 1.6**	**33.24 ± 2.1**	**18.8 ± 1.6**	**10.71 ± 1.4**	**6.52 ± 0.36**	**9.01 ± 0.47**	**9.92 ± 0.95**
Doxorubicin^*a*^	**0.13 ± 0.01**	**0.25 ± 0.02**	**0.24 ± 0.01**	**0.11 ± 0.01**	**0.34 ± 0.02**	**0.55 ± 0.03**	**0.68 ± 0.02**	**0.52 ± 0.03**

^*a*^Positive control.

In the next experiment, we tried to elucidate whether the cytotoxicity caused by Jac-A is from apoptosis. K562 cells were treated with different concentrations of Jac-A and the cytotoxic effects were evaluated by Annexin V and PI dual staining [19]. Annexin V/PI staining in the control group showed a large viable cell population (marked as PI - AV-) and a small amount of early apoptotic (PI - AV+), late apoptotic (PI + AV+), and dead cells (PI + AV-). Jac-A resulted in a shift from viable cells to early and late apoptotic cell population with little change in the dead cell population, especially at the concentration of 10 μM. As shown in Figure 3, flow cytometry analysis showed that Jac-A induced K562 cell apoptosis in a dose-dependent manner. Approximately 2.3% ± 0.9%, 9.5% ± 1.2%, 14.4% ± 2.3%, and 44.7% ± 3.3% PI + AV + cell populations and 1.1% ± 0.7%, 10.2% ± 1.4%, 23.5% ± 3.1%, and 22.1% ± 2.3% PI-AV + cell populations were detected in the 0.1, 1, 5, and 10 μM Jac-A groups, respectively. While no significant apoptotic population was detected in the control group or DMSO group. There was a significance difference in the amount of apoptosis cells in the Jac-A-treated groups compared with the control group. At the same conditions, the positive control (-)-Gossypol showed similar activity of induction apoptosis for K562 cells (Additional file 1: Figure S1). Moreover, Jac-A presented similar activity of apoptosis induction for other leukemia cells HL-60, THP-1 and colon cancer cells LOVO (Additional file 1: Figure S2-S4). After treated with 10 μM of Jac-A, 33.7% ± 3.1% PI + AV + and 29.2% ± 1.4% PI-AV + cell populations were detected in HL-60 cells, and 35.1% ± 2.4% PI + AV + and 27.8% ± 2.1% PI-AV + cell populations were detected in THP-1 cells. However, the activity of apoptosis induction for LOVO cells weaker than for leukaemia cells. Only 17.2% ± 1.6% PI + AV + and 7.89% ± 2.2% PI-AV + cell populations were detected in LOVO cells.

The article "Jacarelhyperol A induced apoptosis in leukaemia cancer cell through inhibition the activity of Bcl-2 proteins" was retracted in 2022. Reasons: duplicated images; original data or images not available; unreliable results or conclusions.

**Figure 3:** **Jac-A caused K562 cell apoptosis.** 10^6^ of K562 cells were treated with different concentrations of Jac-A for 48 h. Cells were then stained with Annexin V-FITC and propidium iodide, and analysed using flow cytometry. Four different cell populations marked as the following: live cell population (PI - AV-), early apoptosis (PI - AV+), late apoptosis (PI + AV+) and dead cells (PI + AV-). Cells were treated with no Jac-A **(A)**, 0.5% DMSO **(B)**, or 0.1, 1, 5, 10 μM/L Jac-A **(C, D, E and F)**. The results are one representative of three independent experiments.

### Jac-A activates caspases cascades

In the intrinsic apoptotic pathway, Bax and Bak, which are regulated by anti-apoptotic Bcl-2 proteins and BH3-only proteins, stimulate the release of cytochrome c from the mitochondrial intermembrane space into the cytosol. Then, cytochrome c induces apoptosome formation, with the activation of caspase-9 as the apical caspase [20]. Caspase-9 further activates the effector caspase-3, which cleaves several hundred cellular proteins, resulting in the characteristic biochemical and morphological features associated with apoptosis, including chromatin condensation, nuclear fragmentation, and externalisation of phosphatidylserine [21]. To elucidate whether cytochrome c fits in Jac-A-induced apoptosis, Jac-A treated K562 cells were lyzed, the cytosol and the mitochondrial membrane portion of the treated cells were obtained through a serial of ultra-centrifugation to probe cytochrome c in both portions using Western blot analysis. As shown in Figure 4A, release of cytochrome c into cytosol was detected in a dose-dependent manner from low as 3 μM of Jac-A at 48 h of treatment. Moreover, we checked the cleavage of caspase-9, caspase-3, and PARP by immunoblotting. As shown in Figure 4B, cleavages of caspase-9, caspase-3, and PARP were detected after K562 cells were treated with Jac-A for 48 h, which is consistent with the previous observation that some inhibitors of antiapoptosis proteins can induce the activation of caspases [22, 23]. In addition, to investigate whether caspases play roles in Jac-A-induced apoptosis of K562 cells, we did another apoptosis assay to examine the effects of a broad-spectrum caspase inhibitor, Z-VAD-FMK on Jac-A-induced apoptosis in K562 cells. K562 cells were first treated with or without different concentrations of Z-VAD-fmk for 4 h, followed by the treatment of Jac-A (10 μM) for 48 h. Cells undergoing apoptosis were measured using by phosphatidylserine (PS) externalization using AnnexinV/FITC in the presence of propidium iodide (PI). As exhibited in Figure 4C, Jac-A-induced apoptosis was inhibited in a concentration dependent manner by the Z-VAD-FMK. These findings suggest that Jac-A-induced apoptosis in K562 cells is partly caspase-dependent.

The article "Jacarelhyperol A induced apoptosis in leukaemia cancer cell through inhibition the activity of Bcl-2 proteins" was retracted in 2022. Reasons: duplicated images; original data or images not available; unreliable results or conclusions.

**Figure 4:** **Jac-A induced caspase-dependent apoptosis in K562 cells. (A)** Cyt c release in Jac-A-induced apoptosis of K562 cells. 10^6^ of K562 cells were treated with different concentration of Jac-A for 48 h. Cytosol and mitochondrial heavy membrane samples were prepared and subjected to immunoblot with anti-Cyt c specific antibodie as described in Materials and methods. The results are one representative of three independent experiments. **(B)** Western blot showing conspicuous cleavage of caspase-3, caspase-9, and PARP in K562 cells treated with Jac-A. K562 cells subjected to protein extract preparation after treated with 0 (control), 3, 6, 12 μM/L Jac-A for 48 h. Then, fifty micrograms extracted protein subjected to Western blot using anti-PARP, PARP, cleaved caspase-9, caspase-9, cleaved caspase-3, caspase-3, and β-actin. The results are one representative of three independent experiments. **(C)** Jac-A-induced apoptosis was inhibited in a concentration dependent manner by the Z-VAD-fmk. K562 cells were first treated with or without different concentrations of Z-VAD-fmk for 4 h, followed by the treatment of Jac-A (10 μM) for 48 h.

### Inhibition of the heterodimerization of antiapoptotic proteins with pro-apoptotic proteins

To confirm that Jac-A binds to anti-apoptotic Bcl-2 family members and competes with binding of pro-apoptotic proteins, co-immunoprecipitation was performed to analyse if these interactions are disrupted by Jac-A. As illustrated in Figure 5, 6 μM of Jac-A treatment started to clearly inhibit the binding of Bcl-x_L_ and Bax. Exposed to 12 μM of Jac-A treatment, little Bcl-x_L_ was seen to bind to Bax. Similarly, less Bcl-2 was observed to bind to Bax at 12 μM of Jac-A treatment than other doses of Jac-A and vehicle control treatment. Moreover, Jac-A also inhibited the binding of Mcl-1 to Bak but the inhibitory effect was presented at 12 μM of Jac-A treatment. These observations demonstrate that Jac-A-induced apoptosis of K562 cells is involved in inhibiting the heterodimerization of antiapoptotic proteins (Bcl-x_L_, Bcl-2, and Mcl-1) with pro-apoptotic proteins (Bax, Bak).

The article "Jacarelhyperol A induced apoptosis in leukaemia cancer cell through inhibition the activity of Bcl-2 proteins" was retracted in 2022. Reasons: duplicated images; original data or images not available; unreliable results or conclusions.

**Figure 5:** **Jac-A inhibited the heterodimerization of antiapoptotic proteins with pro-apoptotic proteins.** Jac-A inhibited the binding between Bax with Bcl-x_L_ or Bcl-2 **(A)** and Bak with Mcl-1 **(B)**. K562 cells were treated with indicated concentrations of Jac-A for 48 h. 150 μg of K562 cell lysates were subjected to co-immunoprecipitation using anti-Bax and anti-Bak antibodies, respectively, further immunoblot with anti- Bcl-x_L_, Bcl-2, Mcl-1, Bax, or Bak antibody, as described in Materials and methods. The results are one representative of three independent experiments.

### Inhibitory effect of Jac-A on K562 cell growth in xenograft mice

To test if Jac-A can inhibit K562 tumour cell growth *in vivo*, we used nude mice that were injected s.c. with K562 cells into the right flank. The K562-bearing mice were randomly divided into four groups (ten mice in each group) and treated with vehicle and Jac-A at a dose of 2, 10, or 50 mg/kg daily for 21 days. As shown in Figure 6A–C, Jac-A dose-dependently inhibited tumor growth. Higher doses of Jac-A had a better inhibitory effect and longer observed survival time (Figure 6D). Interestingly, the body weight of the control group and mice treated with the low-dose of Jac-A were significantly lower than mice from higher dose groups (10 and 50 mg/kg) (Figure 6E). This phenomenon can be attributed to the low toxicity and therapeutic effect of Jac-A. In the process of this experiment, the tumors’ growths of mice from higher dose groups were significantly inhibited and the quality of life better than control group and low-dose group. The absorbed energy from food mainly used for keeping the growth of tumor for mice in control group and low-dose group, which contribute to losing weight. However, this phenomenon improved in higher dose groups. This finding suggests that Jac-A can effectively inhibit the growth of tumor in vivo with low toxicity.

**Figure 6:** **Therapeutic study of Jac-A in the K562-bearing mice (n = 10/group). (A)** Tumour volume plot of K562-bearing mice treated with vehicle or Jac-A at 2, 10, or 50 mg/kg by oral gavage for 21 days. The tumours were measured twice per week. The data are represented as the mean ± SEM. Tumour growth was inhibited significantly after treatment with Jac-A compared with the control group. *, *P* < 0.05; †, *P* < 0.01; ‡, *P* < 0.001 compared with the control group. **(B)** Selected nude mice models of different groups treated with Jac-A or vehicle at day 14 after therapy. **(C)** Sizes of selected tumours harvested from dead nude mice bearing K562 cells from different groups treated with the vehicle or Jac-A. **(D)** Kaplan-Meier survival plot of the K562-bearing nude mice. The survival of the K562-bearing nude mice was prolonged in the Jac-A treated groups compared with control group. **(E)** Body weight plot of the K562-bearing nude mice. The data are represented as the mean ± SEM. *, *P* < 0.05; †, *P* < 0.01; ‡, *P* < 0.001 compared with the control group.

The article "Jacarelhyperol A induced apoptosis in leukaemia cancer cell through inhibition the activity of Bcl-2 proteins" was retracted in 2022. Reasons: duplicated images; original data or images not available; unreliable results or conclusions.

## Discussion

Many anti-cancer drugs have significant side effects, and some cancers are drug resistant [24–26]. Therefore, potential anti-cancer compounds are needed in pharmaceutical development. Natural products, with inherently larger-scale structural diversity than synthetic compounds, are the major resources of bioactive agents and will continue to provide the most candidates for new drug discovery. Many natural product resources have been used as medicine, such as those in traditional Chinese medicine. Active compounds from medicinal plants are generally biologically friendly, because of their clinical use. Here, we identified a new natural Bcl-2 inhibitor Jac-A with potential therapeutic use in murine models of human leukaemia *via* high throughput screening of our in-house NPL and biological testing.

Jac-A, a characteristic constituent of *H. japonicum*, was firstly reported by Kyoko Ishiguro *et al.* and characterized by its inhibitory effect on PAF-induced hypotension [17]. In this work, Jac-A was identified as a new inhibitor of Bcl-2 proteins. We found that Jac-A can compete for binding to BH3 domain of Bcl-2 proteins with proapoptosis proteins in the FP-based binding experiments. This result was confirmed by the co-immunoprecipitation experiment whose results showed Jac-A can inhibit the heterodimerization between antiapoptotic proteins (Bcl-x_L_, Bcl-2, and Mcl-1) with pro-apoptotic proteins (Bax and Bak) in K562 cells. Moreover, Jac-A showed potent activity in inducing the apoptosis of K562 cells. Simultaneously, we found that Jac-A can promote the release of cytochrome c into cytosol and trigger the activation of downstream protein containing caspase-9, caspase-3, and PARP. Additionally, we confirmed that Jac-A-induced apoptosis in K562 cells is partly caspase-dependent based on a broad-spectrum caspase inhibitor Z-VAD-FMK. In the in vivo test, Jac-A also showed a dose-dependentlty inhibition for human K562 cell growth in xenograph tumor mice with low toxicity.

The article "Jacarelhyperol A induced apoptosis in leukaemia cancer cell through inhibition the activity of Bcl-2 proteins" was retracted in 2022. Reasons: duplicated images; original data or images not available; unreliable results or conclusions.

## Conclusions

In summary, we identified the Jac-A, a characteristic component of *H. japonicum*, induces apoptosis in K562 cells by inhibiting the heterodimerization of Bcl-x_L_ /Bcl-2 with Bak, and Mcl-1 with Bax. Together with anticancer activity in vivo, these works not only discovered a new lead compound for cancer therapy with low toxicity, but also provided evidence for using *H. japonicum* as an anti-cancer herb.

## Electronic supplementary material

Additional file 1: Figure S1: (-)-Gossypol caused K562 cells apoptosis. 10^6^ of K562 cells treated with 5 and 10 μM of (-)-Gossypol for 48 h. Cells were then stained with Annexin V-FITC and propidium iodide, and analysed using flow cytometry. Cells were treated with no Jac-A (A), 0.5% DMSO (B), or 5 and 10 μM (-)-Gossypol (C and D).The results are one representative of three independent experiments. **Figure S2.** Jac-A caused HL-60 cells apoptosis. 10^6^ of HL-60 cells treated with 10 μM of Jac-A for 48 h. Cells were then stained with Annexin V-FITC and propidium iodide, and analysed using flow cytometry. Cells were treated with no Jac-A (A), 0.5% DMSO (B), or 10 μM Jac-A (C). The results are one representative of three independent experiments. **Figure S3.** Jac-A caused THP-1 cells apoptosis. 10^6^ of THP-1 cells treated with 10 μM of Jac-A for 48 h. Cells were then stained with Annexin V-FITC and propidium iodide, and analysed using flow cytometry. Cells were treated with no Jac-A (A), 0.5% DMSO (B), or 10 μM Jac-A (C). The results are one representative of three independent experiments. **Figure S4.** Jac-A caused LOVO cells apoptosis. 10^6^ of LOVO cells treated with 10 μM of Jac-A for 48 h. Cells were then stained with Annexin V-FITC and propidium iodide, and analysed using flow cytometry. Cells were treated with no Jac-A (A), 0.5% DMSO (B), or 10 μM Jac-A (C). The results are one representative of three independent experiments. (DOCX 433 KB)

## Abbreviations

Jac-A: Jacarelhyperol A
Bcl-2: B-cell lymphoma 2
NPD: Natural products database
FP: Fluorescence polarisation
MTT: (3-(4,5-dimethylthiazol-2-yl)-2,5-diphenyltetrazolium bromide
TCM: Traditional Chinese medicine
*H. japonicum*: *Hypericum japonicum* Thunb.ex Murray
PAF: Platelet activating factor.
